This article has been retracted.

# Nutrition self-efficacy assessment: designing and psychometric evaluation in a community-dwelling elderly population

**DOI:** 10.1186/s41043-019-0203-3

**Published:** 2019-12-03

**Authors:** Abbas Shamsalinia, Reza Ghadimi, Razieh Torabi Chafjiri, Faezeh Norouzinejad, Ali Pourhabib, Fatemeh Ghaffari

**Affiliations:** 1 Nursing Care Research Center, Health Research Institute, Babol University of Medical Sciences, Babol, I.R Iran; 2 Social Determinants of Health Research center, Health Research Institute, Babol University of Medical Sciences, Babol, I.R Iran; 3 Guilan University of Medical Sciences, Rudsar Shahid Ansari Hospital, Guilan, Rudsar, Iran; 4 Tabriz University of Medical Sciences, Tabriz, I.R Iran

**Keywords:** Community-dwelling elderly population, Self-efficacy, Validity, Reliability, Nutrition, Questionnaire

## Abstract

**Background:**

Awareness of nutrition self-efficacy dimensions can enable healthcare providers to guide their use in screening and providing a context for positive changes such as in promoting a healthy lifestyle and quality care among elderly people.

**Objectives:**

Developing an instrument for assessing nutrition self-efficacy among Iranian elderly population.

**Methods:**

A sequential mixed exploratory design was applied to clarify and determine dimensions of nutrition self-efficacy in a community-dwelling elderly population in two phases. The first phase included a related literature review and a qualitative study. The validity and reliability of the tool were investigated in the second phase. The instrument’s content validity was assessed by experts in nutrition self-efficacy’s field and reliability was determined by internal consistency and construct reliability.

**Results:**

Three factors (adherence efficacy, preventive behaviors, and information effectiveness) and 29 items were obtained after assessing the face, content, and construct validity. The reliability of the nutrition self-efficacy questionnaire (NSEQ) exceeded α > 0.7. Concerning the cumulative percent of the variance, the three factors determined 64.05% of the total variance.

**Conclusions:**

The NSEQ designed in this study, using the background experiences of the elderly living in the community and a review of related texts, and has acceptable reliability and validity. However, the diet self-efficacy questionnaire cannot yet be used as a gold standard, but it can be recommended for use as a measurement of individual diet self-efficacy in a community-dwelling elderly population.

## Highlights

- Nutrition is one of the main aspects of a healthy-oriented lifestyle.
- Exploring the nutrition self-efficacy of older adults can be helpful in a healthcare provider’s design plan for educational and supportive interventions.
- There should be a special questionnaire to explore nutrition self-efficacy among older adults.
- The final version of the NSEQ indicates good validities.
- The NSEQ indicates good homogeneity, stability, and reliability.
- The NSEQ offers a possibility to measure nutrition self-efficacy for healthcare providers.

## Background

Technological advancements have led to an increase in longevity and population-controlling policies have resulted in more elderliness. The elderly population is defined as people aged 60 and over [1].

Elderliness is a sensitive stage of life and its issues and needs to consider it a health priority [2]. Improving and maintaining the health condition in elderliness can not only prevent chronic diseases but can also result in the independence of the elderly in daily routines [3].

Spreading healthy behaviors or a healthy lifestyle, in general, among older adults can result in a decrease in fatalities. Nutritional behaviors are one of the main lifestyle aspects that have a significant impact on the elderly’s health status [4]. Healthy nutrition among older adults is known as an effective behavior for preventing physical or psychological chronic diseases as different scientific papers have mentioned the main role of nutritional behaviors on decreasing coronary artery diseases, decreasing weight and the risk of obesity as well as preventing diabetes and cancers [5, 6]. Nevertheless, aging is accompanied by vast lifestyle changes as the elderly might be diagnosed and treated for chronic diseases as well as faced with a lack of motivation and self-confidence for continuing healthy behaviors [2].

The motivation for following healthy behaviors, such as adhering to diets, meeting the body’s needs or getting fit with new hips, is related to different factors; one is believing in self-abilities to successfully and appropriately following such behaviors [7]. In Iran, nutrition, like other behaviors, is related to the dominant culture and a person’s philosophy [8]. The philosophy that “diseases and death are normal parts of a man’s life” can result in simply coping with daily happenings; such a belief can explain the lack of healthy behaviors among Iranian older adults [8, 9].

One of the most well-known theories on healthy behavior belief change is the social-cognitive learning theory of Bandura (1986), in which perceived self-efficacy is found to be an important construct [10]. Bandura believes that perceived self-efficacy can lead a person toward making health-improving decisions while abandoning harmful ones [11].

The concept of perceived self-efficacy has raised vast discussions among researchers for all generations, especially for older adults, by considering their physiological changes, vulnerabilities and aging conditions [12]. While perceived self-efficacy can be defined as self-judgment regarding self-abilities for doing a specific job and is known as a predicting factor for following health behaviors and accepting health patterns [10], For older adults, self-efficacy has also been related to increased energy, better sleep, and decreased pain and discomfort as well as with overall satisfaction with life [13]. Many studies have mentioned effective interventions to increase perceived self-efficacy in nutrition as an important aspect of the elderly lifestyle [14, 15]. Dieting, weight control, and preventive nutrition can be governed by nutrition self-efficacy beliefs. Nutrition self-efficacy has been shown to be a significant predictor of physical, social and self-evaluative outcome expectancies regarding healthy nutrition [16].

Creating a nutrition self-efficacy instrument for the elderly allows for improving the nutritional behavior of older adults and for healthcare providers to apply appropriate interventions [17]. 

Iran’s population is aging and the proportion of its elderly population in 2050 is likely to reach roughly 20% [18]. Therefore, improving the life quality of this group is one of the healthcare provider’s goals. For this reason, assessing their health condition in different ways using reliable and valid instruments can be helpful in reaching the mentioned goal.

It should be noted that instruments are designed according to a culture’s norms, regulations and healthcare values governing its society. Healthcare professionals believe that culture may influence the application of standardized instruments. Therefore, the translation of an instrument may not have all the necessary criteria for evaluating the nutrition self-efficacy in different cultures [19].

Assessing the self-efficacy for determining older people’s behavioral changes is related to diet management’s future results. Such an assessment needs the evaluation of different self-efficacy factors, even if it might seem challenging. There should be an appropriate instrument recognized and approved to assess the self-efficacy of older adults in each local population. The role of cultural factors is not deniable in older people’s nutritional behavior [20]. The current instruments of diet self-efficacy are not designed for older adults or for older adults with chronic diseases [9, 21]. Nutrition self-efficacy changes vary among elderlies, younger generations, or children as the nutrition needs are different. Healthcare providers are ought to have accessible diet self-efficacy tools in order to be able to determine different aspects of nutrition needs among elderlies. There has been no study yet conducted in Iran based on theories or qualitative approaches to discover the viewpoint of older people’s health expertise in nutrition self-efficacy. Current studies are usually conducted with quantitative approaches to inquire about the self-efficacy of older adults [22, 23] and none of them have used the mixed methods approach as the most complete method to design instruments.

Several self-efficacy instruments for diseases like chronic obstructive pulmonary, asthma, arteries, diabetes, and heart failure are designed and their psychometrics values are tested in the recent two decades [24]. Bandura (2006) has stated that situation, disease, population, or characteristic-based instruments for measuring self-efficacy are needed [11].

Meanwhile, having enough knowledge about the level of nutrition self-efficacy among older adults can provide fundamental information to design more appropriate educational and supportive interventions for first improving self-efficacy and then for improving older people’s lifestyles. The capability of employing health-improving behaviors and adhering to a healthy lifestyle is one of the criteria for classifying an elderly person as an active one [25]; therefore, this study could help healthcare providers to successfully integrate aging into their societies since it presents a questionnaire to screen the nutrition self-efficacy level of older adults. In addition, the results could be helpful to further produce functional research studies to continue exploring the science of nutrition self-efficacy among older adults.

## Objectives

Developing an instrument for assessing the nutrition self-efficacy among Iranian elderly population as well as psychometrically evaluating the reliability and validity of the instrument.

## Methods

This is an inductive-sequential mixed-methods designed study conducted in qualitative and quantitative phases in Guilan and Mazandaran provinces, Iran during 2018. These two provinces are both located in northern Iran and have many cultural beliefs in common. On the other hand, the researchers were at service in these two provinces and accessing the samples was much easier. A deductive-inductive method was used to extract the items for this study. Polit (2006) believes that the use of mixed methods research could provide complementary in research, increase the validity and reliability, and create newer science borders, which show the importance of this method. Toolmaking is one of the functions of mixed methods studies. Polit states that when making a new questionnaire for a health-related issue, the complexity and multi-dimensional aspects of the concept should be explored carefully [26]. This methodological study was conducted in two phases (Fig. 1).

**Fig. 1:** A summary of the study’s method

### Phase one: qualitative study

The qualitative phase is done in two steps: (i) surveying the published literature regarding the self-efficacy concept and its approaches as well as the related instruments for nutrition self-efficacy among older adults and (ii) fieldwork.

#### Review of the international literature

At this stage, researchers checked the data sources of PubMed, Science Direct, ProQuest, OVID, Cinahl, and Scopus without any date filter with relevant keywords, such as elderly, nutrition self-efficacy, lifestyle, nutrition behaviors, and nutrition self-efficacy questionnaire. Textual content analysis was applied to analyze the published literature. The extracted concepts related to nutrition self-efficacy were then turned into items. A list of items was formed. Next, these items were reviewed several times.

#### Semi-structured interviews

The diet self-efficacy data was gathered by semi-structured interviews. There were 15 participants dwelling in the community who could participate if they were interested in participating and they could communicate well. The elderlies who had the inclusion criteria were selected for the interview. These people were able to contact the researcher and were willing to share their views and experiences of the concept of our subject. Researchers invited in-access elderlies like the ones who gathered at retirement centers. Researchers looked for the samples at places in which finding an elderly was easier like mosques, parks, cultural centers, and retirement centers in Mazandaran and Guilan provinces. The elderlies were then asked to fill the questionnaire only if they had satisfaction for participation. The sample was purposively selected to achieve maximum variation (sex, age, education level, etc.) [27]. The interview guiding questions included “explain the concept of nutrition self-efficacy among older adults for me please” and “what are the aspects of nutrition self-efficacy in your mind?” The remaining questions were asked based upon earlier responses. Probing questions like “what do you mean?” or “could you please explain more” were asked as needed. All interviews were face-to-face and were conducted in the researcher’s office at the nursing school.

The sampling was complete when data saturation occurred due to the lack of new categories and subcategories as well as the repeating algorithm of codes. Qualitative content analysis is a conventional method using the Graneheim and Lundman standard that was applied after the data gathering process [28]. The audio records were transcribed and open coding was applied to them. Frequent reviews of the extracted codes helped in finding similarities and differences as well as categorizing them. Finally, the relationships between the categories were explored through data analysis. All extracted codes were then organized into three themes.

### Phase two: quantitative studies

Inductive (items extracted from the participants’ experiences) and deductive (codes extracted from the literature review) methods were used in designing the tool. Researchers prepared a draft of items based on the categories and subcategories formed via the nutrition self-efficacy concept.

### Trustworthiness

Texts were carefully checked by the research team to verify their adherence to the concept. The four criteria of Guba and Lincoln [29]—credibility, dependability, confirmability, and transferability—were applied to check the accuracy of the fieldwork.

### Questionnaire validation

At this stage, the psychometrics of the 67-item questionnaire of nutrition self-efficacy among older people, which was extracted from the literature review and fieldwork was accomplished. The psychometrics of the questionnaire includes two validity and reliability portions.

#### Validity

Ten older adults living in the community were asked to comment on the difficulty, relevancy, and ambiguous levels in face-to-face interviews. A Likert 5-point scale (absolutely important to absolutely unimportant) was used to rank each item, and the older adults were asked to determine the importance of each item according to their experience.

#### Content validity

Five faculty members with sufficient tool designing experience and two nutrition experts were asked to comment on the grammar, wording, allocation, and scaling of the items. The content validity includes Content Validity Index (CVI) and the Content Validity Ratio (CVR):

#### CVR

The Lawshe model (1975) was used to determine the Content Validity Ratio (CVR) [30] in this study. Ten subject matter experts (eight nursing faculty members with tool-making experience and teaching elderly nursing subjects and two nutrition experts) were asked to check the necessity of items.

#### CVI

The Content Validity Index (CVI) was promoted initially by Waltz and Bausell [31]. Ten experts (the same people who helped in the CVR determination) were asked to check if each item fits in the Likert 4-point scale (from absolutely relevant to irrelevant) in order to determine the content validity of each item and to ensure whether the items were designed properly to create the constructs.

#### Convergent and divergent validity

The convergent and discriminant validities of the NSEQ were assessed by Fornell and Larcker approach measuring the average variance extracted (AVE), the maximum shared squared variance (MSV), and the average shared square variance (ASV). For establishing the convergent validity, the AVE had to exceed 0.5, and for the discriminant validity, the MSV and ASV had to be less than the AVE [32].

#### Construct validity

Construct validity was performed by exploratory factor analysis (EFA), which is a way to explore the factors through a variety of variables. In the EFA, the researcher seeks to discover a relatively large set of variables, and the initial assumption is that each variable may be related to any factor. There is no initial theory in this method [33].

#### Reliability

The coefficients of Cronbach’s alpha (α), McDonald’s omega (Ω), and average inter-item correlation (AIC) were estimated to assess the internal consistency (*n* = 388) of the NSEQ. Coefficient’s Ω and α values greater than 0.7 were considered to be acceptable [34].

The construct reliability (CR), which replaces Cronbach’s alpha coefficient in structural equation modeling, was then evaluated, and CR greater than 0.7 were considered acceptable [35]. Also, AIC 0.2 to 0.4 was considered as a good internal consistency [36].

### Setting and samples

The research community includes the older adults living in Guilan and Mazandaran provinces, Iran. Since the acceptable sample size was 5 to 10 samples for each questionnaire item [37], 388 questionnaires were distributed and the data was collected via the conventional method.

### Inclusion and exclusion criteria

The inclusion criteria are as follows. Being older than 60 years of age, being able to read and write, receiving the score of 8 or more in the abbreviated mental test, recognized as independent based on the daily life activities questionnaire [38]. The exclusion criteria are not being under medical treatment or chronic disease treatment follow-up (e.g., diabetes, high blood pressure, coronary artery disease, cerebra vascular accidents, bone and joint diseases).

### Statistical analysis

SPSS version 18.0 was employed for the statistical analyses. The minimally acceptable CVR calculation, based on the modified Lawashe table (2014), was 0.62 [39]. The least acceptable I-CVI score was set to be 0.78; meaning that items with a score less than 0.78 needed to be reformed. We calculated the scale-level content validity index (SCVI) for NSEQ. SCVI under 0.9 was considered appropriate [37]. The acceptable Cronbach’s alpha coefficient and ICC values for the new instrument were found ≥ 0.70. Before starting the EFA, the Kaiser-Mayer-Olkin (KMO) and the Bartlett test was employed [40]. KMO ≥ 0.9 and a significant Bartlett test (≥ 0.05) in factor analysis were acceptable. An EFA using principal components analysis was undertaken to explore the underlying structure of the NSEQ [41, 42]. Variables with factor loadings above 0.4 were extracted [43]. A scree test was used to identify the number of factors [44, 45].

## Results

### First draft of the questionnaire

At the end of the first phase of the study, a pool of 67 items was created. The research team assessed and reviewed the items. Five items were ignored due to their repeating pattern and four were integrated.

### Face and content validity

The results of face and content validity are presented in Fig. 2.

**Fig. 2:** A summary of the instrument development and psychometric evaluation

### Construct validity

First, we conducted a descriptive analysis. The majority of the participants were male (60.1%), married (97.7%), and with the mean age of 66.2 ± 3.2 years (Table 1).

**Table 1:** Demographical characteristics of the study participants (*n* = 388)

Variables	No.		%
Age (mean ± SD,66.2 ± 3.2)			
	60–65	95	24.5
	65–70	248	63.9
	70–75	43	11.1
Gender			
	Female	155	39.9
	Male	233	60.1
Marital status			
	Married	379	97.7
	Widow	6	1.5
	Divorced	1	0.3
	Single	2	0.5
Education level			
	Illiterate	15	3.9
	Primary education	19	4.9
	High school diploma	283	72.9
	Academic education	71	18.3
Employment status			
	Laborer	15	3.8
	Farmer	22	5.7
	Self-employed	151	38.9
	Housewife	100	25.8
	Retired	100	25.8

The standard frequency distributions of responses to each item in the questionnaire were then examined for floor and ceiling effects. There was no missing response and floor or ceiling effect. A NSEQ based on a Likert 5-point scale (5, strongly agree and 1, strongly disagree) was prepared for the exploratory content analysis phase. The KMO value was 0.815. The Bartlett test with the final value of 1711.121 was also considered as significant (*p* < 0.001) meaning that there was enough consistency among the items for factor analysis. Eigenvalues of above 1 and the scree plot were used to determine the number factors in the instrument. The scree plot also confirmed the sufficiency of three factors (adherence efficacy, preventive behaviors, and information effectiveness). The first factor includes 14 items related to adherence efficacy. The most factor load is related to the “I avoid eating foods being in interaction with my drugs” item. The least was the “I can prepare different foods as well as following my own diet” item. The variance ratio calculated for this factor was equal to 56.85. The second factor includes 10 items related to preventive behaviors. The most factor load is related to the “I have enough motivation to buy and prepare healthy foods even when I’m alone” item. The least was the “I pay attention to the nutritional values (e.g., fat, calorie, and minerals) when I want to buy foodstuff” item. The variance ratio calculated for this factor was equal to 60.54. The third factor includes five items related to information effectiveness. The most factor load is related to the “I receive healthy nutrition information from nutrition experts” item. The least was the “I can recognize healthy nutrients when buying them” item. The variance ratio calculated for this factor was equal to 64.05. The three-factor solution explained 64.05% of the total variance based on the scree plot (Table 2). This study does not discuss cross-loadings and deletion of any item. The factor load for each item has been set to 0.4 by the use of component and rotated matrixes (Table 2).

**Table 2:** Results of EFA using rotated component matrix

Domains	Item	Factor 1	Factor 2	Factor 3
Adherence efficacy	1—I follow-up of my diet (weight loss or weight gain up).	.550		
	3—I can follow my age-related diet when I’m in a hurry or busy.	.432		
	11—I prepare appropriate foods for my diet when I eat alone.	.554		
	12—I refuse to eat foods that interaction with my drugs.	.633		
	17—I drink enough amount of water daily according to my physical condition.	.524		
	18—I eat/prepare foods that are rich in calcium and vitamin D according to my physical conditions and needs.	.476		
	20—I adjust my diet according to my digestive problems (e.g., heartburn,dyspepsia, diarrhea, bloating, and anorexia)	.570		
	21—I adjust my diet according to my dental and oral problems (e.g., dry mouth, taste and/or olfaction system defects, and toothless and tooth defects)	.444		
	22- I can prepare different foods as well as following my own diet.	.408		
	26- I can avoid nutrients that increase my blood pressure.	.486		
	4- I adhere to my age-appropriate diet, when I eat at a restaurant.	.595		
	5- I follow my age-related diet when I’m eating at parties.	.458		
	9- I keep my weight steady whenever I got to my ideal body weight.	.432		
	25- I adhere to dietitians’ advice about healthy diet.	.523		
Preventive behaviors	2—I adjust the fat in my diet.		.507	
	7—I ignore eating unhealthy or junk foods (e.g., fast foods, potato chips, and puff )		.448	
	8—I can vegetables and foods rich in fibers according to my physical conditions.		.423	
	14—I can adjust the amount of sugar and sweets in my diet based on my physical conditions.		.517	
	15—I say no to the unhealthy food my family has prepared for me.		.490	
	16—I adjust the amount of salt in my meals.		.449	
	19—I schedule my meals in a way that none of them would be eliminated.		.531	
	23—I have enough motivation to buy and prepare healthy foods, even when I’m alone.		.600	
	27—I buy and eat dairy products (e.g., milk, yogurt, and cheese) based on the level of fat they contain.		.545	
	28—I pay attention to the nutritional values (e.g. fat, Calories and minerals) when I want to buy foodstuff.		.414	
Information effectiveness	6—I know what nutrients a healthy diet is made up of.			.606
	10—I know how to cook foods so their nutritional value would not decrease.			.469
	13—I can recognize healthy foods when buying them.			.409
	24—I receive healthy nutrition information from the dietitian.			.709
	29—I check the accuracy of the nutritional facts presented by friends, family members or media with the nutrition experts.			.443

### What is the scoring procedure for the nutrition self-efficacy questionnaire?

To obtain a mean overall diet self-efficacy, sum scores from all items and divide by 29. To obtain mean scores for individual subscales, sum item scores for each subscale and divide by the number of items.

### Convergent and divergent validity

The results of the convergent and divergent validity of nutrition self-efficacy questionnaire have been inserted into Table 3.

**Table 3:** Convergent, divergent validity (Fornell and Larcker Criterion) and reliability results (*n* = 388)

Dimensions	AVE^a^	MSV^b^	ASV^c^	CR^d^	Ω^e^	^α^ (CI95%)	AIC^f^
Adherence efficacy	0.577	0.334	0.329	0.901	0.801	0.922	0.610
Preventive behaviours	0.514	0.371	0.349	0.912	0.784	0.918	0.331
Information effectiveness	0.636	0.376	0.358	0.913	0.862	0.924	0.449

^a^Average variance extracted

^b^Maximum shared squared variance

^c^Average shared squared variance

^d^Construct reliability

^e^McDonald’s omega coefficient

^α^Cronbach alpha

^f^Average inter-item correlation

### Reliability

Coefficients of Cronbach’s alpha, McDonald’s omega, and CR proved acceptable reliability (> 0.7). The AIC of all factors was also acceptable (Table 3).

### Results of bivariate analysis

Further analysis was conducted to describe the strength and direction of the linear relationships between the factors using Spearman’s rank-order correlation coefficients (Table 4).

**Table 4:** Spearman rank-order correlation coefficient among total factor and individual factors

Factor	1	2	3
	Information effectiveness	Preventive behaviors	Adherence efficacy
1		.719**	.733**
2	.655**		.896
3	.414**	522**	
Total Factor	0.865		

**p< .001 (2-tailed)

## Discussion

This study aimed to evaluate the psychometric properties of the NSEQ. The results of this study showed that NSEQ for community-dwelling elderly population was three factors (adherence efficacy, preventive behaviors, and information effectiveness). According to the reported indices, fitting of the model was considered appropriate. In addition, most loading factors were above 0.4

The items NSEQ are designed for elderlies while all of them can determine diet management needs among this group in this study. Bandura (2006) believes that the items of self-efficacy scales should be able to determine the ability of participants for doing the health behaviors. Items of self-efficacy scales must reflect what man does, but not what he will do. The items should be phrased in terms of can do rather than will do [11].

In this study, the factor loading of all items was significant with the recommended range. Thus, the convergent validity of the scale was confirmed, which is consistent with the results of the original study. The results show an acceptable divergent validity for the factors as the AVE was found to be more than the ASV for each item.

EFA has indicated that the NSEQ contains the three facets of adherence efficacy, preventive behaviors, and information effectiveness. These factors assess 64.05% of the total variance, which is an acceptable number.

The aspects of the questionnaire designed in this study cover the aspects of magnitude, strength and generality in self-efficacy which Bandura (1997) has proposed. “Magnitude” The earliest aspect is self-efficacy beliefs which points to the problems and difficulties that the patient would be ready to face with. “Strength” includes the patients’ conclusions on whether they can overcome a hard behavior or not. “Generality” points to the level of confidence in the patient for doing specific behaviors in different situations and conditions [46].

Based on our findings, the NSEQ has acceptable validity and reliability to be used for inquiring about the nutrition self-efficacy of older adults in a certain community. This questionnaire also had acceptable reliability, and the high Cronbach’s alpha coefficient obtained indicated the good internal consistency of the scale and the correlation between its items. Cronbach’s alpha coefficient was used to check the stability while the coefficient number of 0.7 was proposed as an acceptability level [47].

## Conclusion

Our results support the NSEQ as a reliable and valid instrument for measuring diet self-efficacy of a community-dwelling elderly population. The reliability of this tool needs to be checked in different cultures to verify generalizability.

### Strengths

- Subjects were both men and women.
- There were 13 subject samples for each item, which is an optimal number for factor analysis.
- The NSEQ is already short and fairly easy to complete.
- The NSEQ assesses behavior, motivation, and self-efficacy in a community-dwelling elderly population. The self-efficacy domain covers lifestyle modifications, which are key measures in nutrition management.
- Healthcare providers can use the questionnaire in different places like health centres or older people’s homes as a screening tool for elderly diet self-efficacy.
- The cooperation of nutrition and diet experts as well as faculty members with clinical and tool designing experience beside the older adults of the community resulted in appropriate and highly acceptable validity and reliability for the questionnaire.
- To avoid any ambiguity or misunderstanding of the English translation, the instrument was designed in Farsi (Persian) but translated into English at the same time with the manuscript and as we used to, two bilingual researchers and academics helped us with back-translation which showed a perfect match.

### Limitations

- The lack of related studies in Iran and the absence of similar tools in Iran and other countries.
- Although this questionnaire has good validity, cultural differences, language, and educational level between different regions of the world and elderly people living in Iranian society may affect the validity.
- This study was conducted in a district of northern Iran that limits the generalizability of the results. The researchers tried to minimize this limitation by using the maximum variation in interviews.
- Inclusion criteria can limit the use of the questionnaire presented in this study.
- One of the NSEQ advantages is that it only requires 20 min to be completed. However, it might not be suitable for some studies as a questionnaire with less items cannot completely explore the complex construction of the diet self-efficacy among older adults.
- A self-report tool can be influenced by the psychological variables of the samples.

## Supplementary information

**Additional file 1.** S1 File. NSEQ-29_Persian version.

**Additional file 2.** DSEQ-29_ English version.

## Data Availability

Data generated or analyzed during this study are included in this published article and are available from the corresponding author on reasonable request.

## Abbreviations

CVI: Content Validity Index
CVR: Content Validity Ratio
EFA: Exploratory factor analysis
ICC: Intraclass correlation coefficient
KMO: Kaiser-Meyer-Olkin
NSEQ: Nutrition self-efficacy questionnaire
